This article has been retracted.

# Piceatannol inhibits pyroptosis and suppresses oxLDL-induced lipid storage in macrophages by regulating miR-200a/Nrf2/GSDMD axis

**DOI:** 10.1042/BSR20201366

**Published:** 2020-09-16

**Authors:** Zhongyuan Mu, Hongling Zhang, Peng Lei

**Affiliations:** 1 Heart Center, The First Hospital of Lanzhou University, Lanzhou, Gansu, China; 2 Gansu Provincial Clinical Research Center for Cardiovascular Diseases, Lanzhou, Gansu, China; 3 Key Laboratory for Cardiovascular Diseases of Gansu Province, Lanzhou, Gansu, China; 4 Department of Gastroenterology, The First Hospital of Lanzhou University, Lanzhou, Gansu, China

**Keywords:** atherosclerosis, GSDMD, miR-200a, nrf2, piceatannol, pyroptosis

## Abstract

As a major bioactive compound from grapes, piceatannol (PIC) has been reported to exert anti-atherosclerotic activity in various studies. Nevertheless, the mechanism underlying the effect of piceatannol against atherosclerosis (AS) is elusive. Our study identified miR-200a/Nrf2/GSDMD signaling pathway as critical mediators in the effect of piceatannol on macrophages. In the present study, we confirmed that treatment of piceatannol repressed the oxLDL-induced lipid storage in macrophages. Compared with control group, piceatannol inhibited TG storage and the activity of caspase1. It is noting that in response to oxLDL challenge, piceatannol abated the pyroptosis in RAW264.7 cells, with a decreased expression of caspase1, gasdermin D (GSDMD), IL-18, IL-1β and NLRP3. Moreover, we investigated the role of microRNA (miR)-200a/Nrf2 signaling pathway in the effect of piceatannol. The results declared that after transfection of si-miR-200a or si-Nrf2 plasmids, the effects of piceatannol on macrophages were converted, including lipid storage and pyroptosis. Importantly, si-miR-200a plasmid reduced the expression of nuclear factor erythroid 2-related factor 2 (Nrf2), indicating that miR-200a acted as an enhancer of Nrf2 in macrophages. Collectively, our findings demonstrate that piceatannol exerts anti-atherosclerotic activity on RAW264.7 cells by regulating miR-200a/Nrf2/GSDMD signaling. The present study is the first time to identify miR-200a as a candidate target in AS and declared an association between miR-200a and pyroptosis, which provides a novel therapy for the treatment of AS.

## Introduction

As a chronic vascular disease, atherosclerosis (AS) is currently seriously affecting human health. AS is associated with multiple risk factors, such as hyperlipidemia, hypertension, diabetes, and smoking [1]. A dysfunction of macrophage is regarded as the critical step in the development of AS. In the progression of AS, the formation of plaque necrosis is promoted by the death of lesional macrophages and defective phagocytic clearance of the dead cells [2]. Pyroptosis is a highly inflammatory programmed cell death and also an important form of innate immune response during infections and tissue damages [3,4]. Previous studies suggest that pyroptosis plays an important role in advanced lesional macrophage death. In the process of macrophage death, two signals were required to up-regulate pro-IL-1β and to induce NLRP3-mediated maturation of IL-1β [5]. Interaction of NLRP3 with ASC recruits pro-CASP1, and then cleaves and releases mature IL-1β via pores formed by gasdermin D (GSDMD) [6].

As a natural phenolic compound with similar chemical structure to resveratrol, piceatannol (PIC) is believed to exert beneficial effects similar to resveratrol [7]. It has been well known that piceatannol showed various cardioprotective activities such as inhibition of low-density lipoprotein cholesterol oxidation, inhibition of platelet aggregation, and mediation of cardiac cell function [8]. Several researches revealed that piceatannol exhibits anti-inflammatory effects on macrophages [9]. For example, piceatannol inhibited LPS-induced proinflammatory gene expression and synthesis of nitric oxide (NO), tumor necrosis factor-a (TNF-a), and interleukin-6 (IL-6) in RAW264.7 macrophages. Moreover, piceatannol acted as an SYK inhibitor, and completely blocked oxLDL-induced MHC-II and MAPK8 expression in BMDM, indicating a decrease in autophagy, which provided new insights into the therapy of AS [10]. Although, piceatannol inhibited the proliferation and migration of vascular smooth muscle cells to protect against AS [11], little is known about the role of pyroptosis inhibited by piceatannol on macrophages in the protection of AS.

As one of the most essential transcription factors, nuclear factor erythroid 2-related factor 2 (Nrf2) exerts antioxidant, anti-apoptotic, and anti-inflammatory effects by interacting with multiple signaling pathways [12,13]. It has been declared that in response to an oxidative stress, Nrf2 transferred to the nucleus and bind to the antioxidant response element (ARE), which increased the expression of the phase II antioxidant enzymes [14]. Importantly, in diabetic cardiomyopathy, piceatannol alleviates inflammation and oxidative stress by regulating the Nrf2/HO-1 and NF-kB pathways. Knockdown of Nrf2 suppressed PIC-induced enhancement of HO-1 expression and abolished the anti-inflammatory effects of PIC [15]. Moreover, piceatannol attenuates homocysteine-induced apoptosis, oxidative stress, and endoplasmic reticulum stress via Nrf2-dependent HO-1 expression in endothelial cells [16]. Notably, there is a cross-talk between Nrf2 and microRNA (miRNA or miR) in cell pyroptosis. For instance, miR-181 inhibits the activation of SIRT1/PGC-1a/Nrf2 pathway, leading to an increase in cell pyroptosis in human neuroblastoma SH-SY5Y cells [17]. However, the role of Nrf2 and miRNA under the treatment of piceatannol in macrophages have not been fully elucidated.

In the present study, we found that piceatannol attenuated the lipid accumulation in macrophages in response to oxLDL challenge, which was associated with decreased level of pyroptosis. It is noting that up-regulation of miR-200a/Nrf2 signaling was also identified in the study. Additionally, we explored the effect of miR-200a/Nrf2 signaling on piceatannol treatment to protect against lipid accumulation in macrophages. Our study may provide new insights into the therapy of AS.

## Materials and methods

### Cell culture and chemicals

RAW264.7 macrophage cells were kindly gifted by Dr. Li from Peking University in China, and cultured in RPMI 1640 medium, which contained 10% FBS (P30-3301; Pan) and 1% penicillin–streptomycin (15140-122; Gibco). Cells were cultured in 5% CO_2_ under a water-saturated atmosphere in a cell incubator at 37°C. The *trans*-isomer of piceatannol (PIC) was purchased from Sigma–Aldrich, St. Louis, MO, U.S.A. (P0453-5MG; Sigma). DMSO (276855, Sigma) was used as the negative control.

### Cell transfection

The si-Nrf2 plasmid, miR-200a mimic, and their negative controls were procured from GenePharma (Shanghai, China). The RAW264.7 cells were cultured in six-well plates at a density of 1 × 10^7^ cells/ml for 24 h. Lipofectamine 2000 reagent (11668-027, Invitrogen) was used for transfection according to the manufacturer’s instructions. After transfection for 48 h, cells were collected for further researches.

### Caspase1 activity assay

RAW264.7 cells (1 × 10^6^ cells/well) were cultured in 24-well microplates, and then seeded overnight at 37°C in a 5% CO_2_ incubator. Furthermore, the cells were treated with PIC (30 μM) for 48 h. All protein was extracted by using cell lysis buffer (R0020, Solarbio) from the macrophages. After that, centrifugation was used to clear lysates, following with a measurement of protein concentration by BCA protein assay kit (P1511-1, Applygen). Caspase1 activity kit (BC3810, Solarbio) was used according to the manufacturer’s instructions. The plate reader was used to determine the absorbance values at 405 nm. The activity levels were expressed compared with the control group.

### Oil Red O staining

RAW264.7 cells were stained in a 60% Oil Red O working solution (G1262, Solarbio) for 30 min to examine intracellular lipid accumulation. Commercial kits (BC0620, BC1985; Solarbio) were used to measure the contents of total cholesterol (TC) and triglyceride (TG) in the macrophages, according to the manufacturer’s instructions.

### Relative LDH release

First, cells were centrifuged at 1000 rpm for 2 min. Subsequently, according to the manufacturer’s instructions, relative LDH release was determined using a commercial kit (BC0685, Solarbio). The absorbance of samples was assessed at 490 nm using a microplate reader.

### Western blot analysis

After all treatment, RAW264.7 cells were lysed in RIPA lysis buffer (R0020, Solarbio), containing 1% protease inhibitor cocktail (B14001; Bimake) and 1% phosphatase inhibitor (B15001; Bimake). The protein concentration of lysate was determined by using BCA Assay Kit (P1511-1, Applygen). Twenty micrograms of protein was isolated using 10% SDS/PAGE and electro-transferred to PVDF membranes (IPVH00010; Millipore). The membranes were blocked by TBST containing 5% milk for 2 h at room temperature, and probed with various primary antibodies at 4°C overnight. After being washed with TBST at intervals of 10 min, membranes were incubated with HRP-conjugated secondary antibodies for 2 h at room temperature. After washing for five times, the immunoreactive bands were visualized using Clarity Western ECL Substrate (170-5060; Bio-Rad). The protein bands were visualized with a Bio-Rad System (Bio-Rad, Hercules, CA, U.S.A.). Actin served as a loading control.

### Antibodies

Antibodies against caspase1 (A16792), actin (AC026) were obtained from ABclonal (Wuhan, China). Antibodies specific for IL-1β (ab9722), IL-18 (ab191152), GSDMD (ab210070), NLRP3 (ab263899), Nrf2 (ab92946) were purchased from Abcam (Cambridge, MA, U.S.A.). The dilution ratio for all primary antibodies was 1:2000. The secondary antibodies used in the present study were peroxidase AffiniPure goat anti-rabbit-IgG (H+L) (BF03008X) and goat anti-mouse-IgG (H+L) (BF03001X) obtained from Biodragon (Beijing, China). Secondary antibodies were used at 1:5000 dilution.

### Real-time PCR assay

Briefly, TRIzol reagent (15596-026; Invitrogen) was used to isolate total RNA from RAW264.7 cells. The extraction of RNA was conducted on the basis of the manufacturer’s instructions, along with the transcription of RNA samples into cDNA employing a Transcriptor First-Strand cDNA Synthesis Kit (04896866001; Roche). The ABI-Quant Studio 5 system and the SYBR Green PCR Master Mix Reagent Kit (TransGen, Beijing, China) were used to quantify the PCR amplification products. The mRNA expression levels of the target genes were normalized to β*-actin* expression. The primer pairs used in the present study are listed in Supplementary Table S1.

### Statistical analysis

Experimental data were expressed by mean ± SEM. Using GraphPad Prism 8.0 software (GraphPad Software, Inc., San Diego, CA) to analyze differences among the various treatment groups by two-tailed Student’s *t* test or one-way ANOVA. Data from all studies were collected in a blinded fashion. No data were excluded when performing the final statistical analysis. The difference was statistically significant at *P*<0.05.

## Results

### Effects of piceatannol on the lipid storage and caspase1 activity in macrophages

To determine the effect of PIC (Figure 1A) on oxLDL-induced lipid storage in macrophages, macrophages RAW264.7 were treated with oxLDL (80 mg/l) for 24 h in the absence or presence of PIC (30 μM). First, we used Oil Red O staining to detect the lipid content. As shown in Figure 1B, oxLDL induced an increase in lipid storage in macrophages, but the PIC administration revised the high level of lipid accumulation. Moreover, we measured the content of TG and TC in macrophages after PIC treatment. Similar to the results of Oil Red O staining, oxLDL treatment led to increased TG and TC levels. However, PIC administration markedly decreased the content of TG and TC in macrophages (Figure 1C,D). Then, we found that PIC was able to convert the elevation of caspase1 activity induced by oxLDL in macrophages (Figure 1E). Collectively, these data suggested that PIC could inhibit oxLDL-induced lipid accumulation and caspase1 activity in macrophages.

**Figure 1:** Effects of piceatannol on the lipid storage and caspase1 activity in RAW264.7 cells (**A**) Chemical structure of piceatannol. (**B**) Representative images by using Oil Red O staining after administration of piceatannol. The experiments were repeated three times. (**C,D**) Analysis of TG and TC content in macrophages. *P<0.05, ***P<0.001. The experiments were repeated three times. (**E**) Analysis of the caspase1 activity after piceatannol treatment. *P<0.05, ***P<0.001. The experiments were repeated four times.

### Effects of piceatannol on the pyroptosis of macrophages after oxLDL exposure

Furthermore, we speculated whether PIC treatment affected the level of pyroptosis. Hence, real-time PCR analysis was carried out to detect the level of pyroptosis. As expected, the results showed that PIC inhibited pyroptosis of macrophages when exposed to oxLDL. In mRNA level, GSDMD and caspase1 expression were down-regulated after PIC administration as compared with the cells without PIC treatment (Figure 2A). We also detected the expression level of NLRP3, IL-18, and IL-1β, which was positively associated with GSDMD [18,19]. We observed that the expression of NLRP3, IL-18, and IL-1β were both decreased after administration of the PIC (Figure 2A). Moreover, we used Western blot to assess the protein level related to pyroptosis. The results indicated that PIC attenuated oxLDL-induced high level of GSDMD, caspase1 p10, NLRP3, cleaved IL-18, and IL-1β (Figure 2B–D). In addition, PIC treatment blocked the up-regulation of LDH release activity (Figure 2E), which indicated an improvement of membranolysis and cell death of RAW 264.7 cells. The results suggested that PIC was an effective molecule for suppressing pyroptosis in macrophages.

**Figure 2:** Effects of piceatannol on the pyroptosis of macrophages after oxLDL challenge (**A**) qPCR analyses of the relative mRNA levels of caspase1, GSDMD, IL-18, IL-1β, and NLRP3 on RAW264.7 cells after piceatannol treatment. Gene expression was normalized to β-actin mRNA level. *P<0.05, **P<0.01, ***P<0.001. The experiments were repeated four times. (**B–D**) Representative Western blot analysis (B) and quantification (C,D) of caspase1, GSDMD, NLRP3, cleaved IL-18 and IL-1β protein on RAW364.7 cells after piceatannol administration. Protein expression was normalized to β-actin levels. *P<0.05, **P<0.01, ***P<0.001. The experiments were repeated three times. (**E**) Analysis of LDH release after piceatannol treatment. **P<0.01, ***P<0.001. The experiments were repeated four times. Abbreviation: qPCR, real-time PCR.

### Role of Nrf2 on the effects of piceatannol on macrophages in response to oxLDL exposure

It has been well known that Nrf2 was up-regulated in the effect of PIC against AS. Therefore, we postulated that PIC might target Nrf2 to modulate pyroptosis in macrophages. Notably, we found that both in mRNA and protein level, PIC up-regulated Nrf2 expression in macrophages (Figure 3A,B). Moreover, PIC treatment promoted the expression of HO-1, GCLC, and CD36, which were the downstream genes of Nrf2 (Figure 3C). These results supported that PIC significantly enhanced the Nrf2 expression and its activity. Furthermore, anti-Nrf2 plasmids were transfected into macrophages. Then, we examined the lipid storage in macrophages after PIC treatment and plasmid transfection. We found that when exposed to oxLDL, the anti-Nrf2 plasmids were able to convert the low lipid accumulation induced by PIC in macrophages (Figure 3D). Moreover, TG and TC content were also increased after plasmid transfection (Figure 3E,F). To further analyze the role of Nrf2 in the effect of PIC in macrophages, we detected the level of pyroptosis after the PIC administration and the transfection of anti-Nrf2 plasmids. Notably, by using real-time PCR and Western blot assay, anti-Nrf2 plasmids significantly reversed the level of pyroptosis induced by PIC as compared with vehicle group, with an up-regulation of the expression of caspase1 p10, GSDMD, NLRP3, cleaved IL-18 and IL-1β (Figure 3G,H). In addition, si-Nrf2 plasmid abated the PIC-induced amelioration of LDH release activity (Figure 3I). The results demonstrated that Nrf2 plays an important role in the pyroptosis regulated by PIC in macrophages.

**Figure 3:** Role of Nrf2 on the effects of piceatannol on macrophages when exposed to oxLDL (**A**) qPCR analyses of the relative mRNA levels of Nrf2 on RAW264.7 cells after piceatannol treatment. ***P<0.001. The experiments were repeated four times. (**B**) Representative Western blot analysis of Nrf2 protein on RAW264.7 cells after piceatannol administration. Protein expression was normalized to β-actin levels. The experiments were repeated three times. (**C**) The mRNA levels of HO-1, GCLC, and CD36 after piceatannol treatment. **P<0.01, ***P<0.001. The experiments were repeated four times. (**D**) Representative images by using Oil Red O staining after plasmid transfection. The experiments were repeated three times. (**E,F**) Analysis of TG and TC content in macrophages. **P<0.01, ***P<0.001. The experiments were repeated three times. (**G**) Representative Western blot analysis of caspase1, GSDMD, NLRP3, cleaved IL-18 and IL-1β protein after plasmid transfection. Protein expression was normalized to β-actin levels. The experiments were repeated three times. (**H**) qPCR analyses of the relative mRNA levels of caspase1, GSDMD, IL-18, IL-1β, and NLRP3 after transfection of si-Nrf2 plasmid. Gene expression was normalized to β-actin mRNA level. *P<0.05, **P<0.01, ***P<0.001. The experiments were repeated four times. (**I**) Analysis of LDH release after plasmid transfection of si-Nrf2. *P<0.05, **P<0.01. The experiments were repeated four times. Abbreviation: qPCR, real-time PCR.

### Role of miR-200a on the effects of piceatannol on macrophages in response to oxLDL exposure

Previous studies provided a robust evidence to support a cross-talk between Nrf2 and miR-200a [20,21]. Hence, we speculated that miR-200a could act as an upstream of Nrf2, and was closely involved in the effect of PIC in macrophages. Initially, we demonstrated that PIC increased miR-200a level in RAW264.7 cells (Figure 4A). To further explore the role of miR-200a in PIC-mediated pyroptosis, we knocked down miR-200a expression with si-miR-200a plasmid (Figure 4B). We found that in response to oxLDL exposure, knockdown of miR-200a completely blocked the inhibition of lipid accumulation after treatment with PIC, with increased content of TG and TC in macrophages (Figure 4C–E). Moreover, we detected the level of pyroptosis after transfection of si-miR-200a plasmid. The results showed that the LDH release activity was increased after plasmid transfection (Figure 4F). In addition, compared with vehicle control, plasmid transfection led to an increased expression of caspase1 p10, GSDMD, NLRP3, cleaved IL-18 and IL-1β both in mRNA and protein level (Figure 4G,H). Notably, knockdown of miR-200a converted the high protein expression of Nrf2 induced by PIC treatment, suggesting that miR-200a was the upstream of Nrf2. Combined, we concluded that PIC inhibited pyroptosis in macrophages by regulating miR-200a/Nrf2 pathway.

**Figure 4:** Role of imR-200a on the effects of piceatannol on macrophages in response to oxLDL exposure (**A**) qPCR analyses of the relative mRNA levels of miR-200a on RAW264.7 cells after piceatannol treatment. *P<0.05, ***P<0.001. The experiments were repeated four times. (**B**) The mRNA levels of miR-200a after transfection of si-miR-200a plasmids. ***P<0.001. The experiments were repeated four times. (**C**) Analysis of TG content in macrophages. *P<0.05, ***P<0.001. The experiments were repeated three times. (**D**) Representative images by using Oil Red O staining after plasmid transfection. The experiments were repeated three times. (**E**) Analysis of TC content in macrophages. *P<0.05, ***P<0.001. The experiments were repeated three times. (**F**) Analysis of LDH release after plasmid transfection of si-miR-200a. *P<0.05, **P<0.01. The experiments were repeated four times. (**G**) qPCR analyses of the relative mRNA levels of caspase1, GSDMD, IL-18, IL-1β, and NLRP3 after transfection of si-miR-200a plasmid. Gene expression was normalized to β-actin mRNA level. *P<0.05, **P<0.01, ***P<0.001. The experiments were repeated four times. (**H**) Representative Western blot analysis of Nrf2, caspase1, GSDMD, NLRP3, cleaved IL-18 and IL-1β protein after plasmid transfection. Protein expression was normalized to β-actin levels. The experiments were repeated three times. Abbreviation: qPCR, real-time PCR.

## Discussion

AS is a chronic cardiometabolic disease, and remains the leading cause of deaths around the world [22]. Due to unapparent clinical manifestation, AS is commonly diagnosed only after a cardiovascular event such as a myocardial infarction or stroke, which leads to an extremely high mortality [23]. Hence, it is necessary to investigate the potential drug and explore the underlying molecular mechanisms on AS. As a natural compound extracted from grapes, it has been well shown in various researches that PIC can protect against AS [10,24]. However, the specific molecular mechanism has not been evaluated yet. In the study, we investigated the mechanism underlying the anti-atherogenic effects of PIC. The results provide robust evidence that modulation of miR-200a/Nrf2/GSDMD is closely involved in the effect of PIC against AS, which provides new insights into the clinical therapy of AS.

As a novel form of cell death, pyroptosis is uniquely dependent on caspase1 which is not involved in apoptosis [25,26]. It has been well demonstrated that various natural compounds exerted anti-atherogenic effects by inhibiting pyroptosis, such as nicotine [27], sinapic acid [28], melatonin [29]. Here, we found that PIC attenuated oxLDL-induced lipid storage by inhibiting pyroptosis in RAW264.7 cells. OxLDL is an important biomarker of cardiovascular diseases. In patients with chronic metabolic disorders, the oxLDL levels are significantly increased [30,31]. Moreover, previous study has reported that in apolipoprotein E knockout mice, plasma oxLDL was obviously elevated during the progression of AS [32]. The proatherogenic properties of oxLDL attribute to its cytotoxicity toward all vascular cells and macrophages [33,34]. In atherosclerotic lesions, enhanced macrophage death promotes the formation of necrotic cores, which is a representative feature of advanced atherosclerotic plaques [35]. Consistent with these observations, we found an increase in lipid storage in macrophages after oxLDL exposure, which is converted by PIC treatment. Notably, the results declared that PIC attenuated oxLDL-induced pyroptosis in RAW264.7 cells, which is similar to Guo et al.’s findings that oxLDL potently enhanced pyroptosis in macrophages [36]. Furthermore, we confirmed a down-regulated expression of NLRP3, IL-18, and IL-1β after PIC treatment. NLRP3 is the sensor of NLRP3 inflammasome which also contains an adaptor (ASC; also known as PYCARD) and an effector (caspase1). Formation of the inflammasome activates caspase1, and in turn cleaves pro-IL-1β, pro-IL-18 and GSDMD, which promotes GSDMD to insert into the membrane and form pores and inducing pyroptosis [37]. Enhanced activation of caspase1 contributes to a high level of IL-1β and IL-18 [38,39]. In this study, the results showed that the caspase1 expression was obviously down-regulated after PIC treatment, which led to a decrease in IL1b and IL18 expression. These results robustly support that PIC exerts anti-atherosclerotic activity by regulating pyroptosis in macrophages.

Furthermore, we explored the role of miR-200a/Nrf2 signaling pathway in the effect of PIC on macrophages. As a master regulator of cytoprotective genes, Nrf2 is known for its antioxidant and anti-inflammatory properties [40]. According to previous studies, Nrf2 is closely involved in the regulation of pyroptosis. For instance, in vascular endothelial cells, knockdown of Nrf2 abrogated the DHM-medicated improvement in ROS generation and PA-induced pyroptosis [40]. Moreover, erythropoietin rescues primary rat cortical neurons from pyroptosis by up-regulating Erk1/2-Nrf2/Bach1 signaling pathway [41]. In our study, we found that PIC treatment promoted the expression of Nrf2 and its typical targets, such as HO-1, GCLC, and CD36, which suggested an enhancement of Nrf2 activation. Notably, several reports have demonstrated that Nrf2 contributes oxLDL uptake by inducing CD36 [42]. In this study, we observed an increase in CD36 expression in Nrf2-dependent manner after PIC treatment, which might contribute to an up-regulation of oxLDL uptake. However, PIC can also act as a SYK inhibitor to induce autophagy in RAW264.7 cells [10], which has been proved to play an important role in the clearance of oxLDL. Notably, an inhibition of pyroptosis induced by VX-765 improves the lipid storage in vascular smooth muscle cells [43]. Therefore, the PIC-induced reduction in lipid accumulation in macrophages may mainly attribute to the inhibition of pyroptosis and the induction of autophagy. In further research, we will detect the proportion of these two pathways in macrophages and explore other potential mechanism after PIC treatment.

It is worth noting that as an upstream of Nrf2, miR-200a has been reported to regulate the Nrf2 activation. Elevated expression of miR-200a inhibits Keap1 and up-regulates Nrf2 nuclear translocation, which results in a decrease in ROS production in human adult cardiomyocyte line in response to hypoxia exposure [44]. It has been proved that aberrant miR-200a expression targets to Keap1 and then inhibits Nrf2 antioxidant pathway [45]. Similar to previous studies, we found that PIC increased the expression of miR-200a and Nrf2 in oxLDL-treated macrophages. The level of lipid storage was converted after transfection of si-miR-200a or si-Nrf2 plasmids. In addition, the transfection of these two plasmids also inhibited the PIC-mediated pyroptosis. Importantly, the results revealed that compared with the group with single treatment of PIC, si-miR-200a plasmids reduced the Nrf2 expression, suggesting that miR-200a was also regarded as an enhancer of Nrf2 in the anti-atherogenic effect of PIC in macrophages.

Collectively, we identified PIC as a potential candidate for the treatment of AS by regulating miR-200a/Nrf2/GSDMD signaling pathway. When exposed to oxLDL, the PIC administration inhibited pyroptosis and lipid accumulation in macrophages by up-regulating miR-200a and Nrf2. Transfection of si-miR-200a or si-Nrf2 plasmids reversed the effect induced by PIC. It is the first time to declare that PIC alleviates AS by inhibiting pyroptosis, and demonstrated an association between miR-200a and pyroptosis. The present study provides evidences to support PIC to be regarded as a strong option for therapy of AS.

## Supplementary Material

Supplementary Table S1

## Abbreviations

AS: atherosclerosis
BMDM: bone-marrow-derived macrophage
CASP1: caspase1
GCLC: glutamatecysteine ligase catalytic subunit
GSDMD: gasdermin D
HO-1: heme oxygenase 1
HRP: horse radish peroxidase
Keap1: kelch-like ECH-associated protein 1
LDH: lactate dehydrogenase
LPS: lipopolysaccharide
miR/miRNA: microRNA
NLRP3: NLR family pyrin domain containing 3
Nrf2: nuclear factor erythroid 2-related factor 2
oxLDL: oxidized low-density lipoprotein
PA: palmitic acid
PGC-1a: peroxisome proliferator-activated receptor gamma coactivator 1-alpha
PIC: piceatannol
ROS: reactive oxygen species
SIRT1: sirtin1
TC: total cholesterol
